# Development and External Validation of a Nomogram for Predicting Overall Survival in Stomach Cancer: A Population-Based Study

**DOI:** 10.1155/2021/8605869

**Published:** 2021-09-24

**Authors:** Haonan Ji, Huita Wu, Yu Du, Li Xiao, Yiqin Zhang, Qiuhua Zhang, Xin Wang, Wenfeng Wang

**Affiliations:** ^1^Department of Oncology, Zhongshan Hospital Affiliated to Xiamen University, Xiamen, China; ^2^School of Science, Shanghai Institute of Technology, Shanghai 201418, China; ^3^International Academy of Visual Art and Engineering, London E16 1AH, UK; ^4^Interscience Institute of Management and Technology, Bhubaneswar 752054, India; ^5^RCEECA, Chinese Academy of Sciences, Urumqi 830011, China

## Abstract

**Objective:**

The study was to develop and externally validate a prognostic nomogram to effectively predict the overall survival of patients with stomach cancer.

**Methods:**

Demographic and clinical variables of patients with stomach cancer in the Surveillance, Epidemiology, and End Results (SEER) database from 2007–2016 were retrospectively collected. Patients were then divided into the Training Group (*n* = 4,456) for model development and the Testing Group (*n* = 4,541) for external validation. Univariate and multivariate Cox regressions were used to explore prognostic factors. The concordance index (C-index) and the Kolmogorov–Smirnov (KS) value were used to measure the discrimination, and the calibration curve was used to assess the calibration of the nomogram.

**Results:**

Prognostic factors including age, race, marital status, TNM stage, surgery, chemotherapy, grade, and the number of regional nodes positive were used to construct a nomogram. The C-index was 0.790 and the KS value was 0.45 for the Training Group, and the C-index was 0.789 for the Testing Group, all suggesting the good performance of the nomogram.

**Conclusion:**

We have developed an effective nomogram with ten easily acquired prognostic factors. The nomogram could accurately predict the overall survival of patients with stomach cancer and performed well on external validation, which would help improve the individualized survival prediction and decision-making, thereby improving the outcome and survival of stomach cancer.

## 1. Introduction

Stomach cancer is a kind of malignant tumor with high invasiveness and heterogeneity, which is a global health problem [1]. It remains the fifth most common cancer and the third leading killer of cancer-related deaths worldwide despite the decreasing trend of new morbidity and mortality [2, 3]. It is estimated that about 783,000 people died of stomach cancer in 2018, and 769,000 died in 2020 globally [2, 4]. There will be approximately 26,560 new cases of stomach cancer and 11,180 deaths in the United States in 2021 according to the American Cancer Society (https://www.cancer.org/cancer/stomach-cancer/about/key-statistics.html). The prognosis of early stomach cancer is relatively good, and the 5-year survival rate is about 69–82% [5]. Despite advances in radical surgical techniques and perioperative chemotherapy, the survival rate of patients with advanced stomach cancer remains poor. The 5-year overall survival of them is mostly under 50% [6]. Herein, it is of great significance to identify independent prognostic factors of stomach cancer for the better treatment and prognosis of cancer.

Some known demographic and clinicopathological variables affect the survival of gastric cancer patients [3, 7–10], and a comprehensive model based on these factors needs to be developed to predict individual survival. Several previous studies have proposed nomograms predicting survival of patients with stomach cancer [11–13]. Kim et al. developed prognostic nomograms based on several clinicopathological variables, which can independently predict the overall survival of advanced gastric cancer patients (unresectable or metastatic gastric cancer after combined cytotoxic chemotherapy as first-line treatment) [11]. Besides, another study showed a prognostic nomogram utilizing the systemic immune inflammation index to predict the overall survival of patients with stomach cancer after operation [12]. Although the evaluation indicators of these nomogram models were great, most of the studies were based on patients who received surgery, or patients with a specific stage of disease, such as patients in advanced stages or after radiotherapy and chemotherapy. Later, the prognostic nomogram for this research included nonresection patients, but it only used clinical prognostic factors [13].

In the present study, we aimed to develop a prognostic nomogram, which included patients with or without surgery and other treatments, using easy-to-collect demographic (age, race, and marital status) and clinicopathological variables (TNM stage, surgery, chemotherapy, grade, and the number of regional nodes positive). The prognostic nomogram may help clinicians more accurately predict the overall survival of patients with stomach cancer, thereby optimizing the treatment selection and improving the prognosis of cancer.

## 2. Methods

### 2.1. Study Population

The SEER database is the most comprehensive registry of cancer incidence and survival in the United States and representative of 34.6% of the US population. It complies with patient-level data collected from 18 geographically diverse populations that represent rural, urban, and regional populations [10]. In the present study, 10,430 patients diagnosed with stomach cancer in the SEER database from 2007 to 2016 were retrospectively reviewed. After screening, a total of 1,433 patients were excluded for incomplete clinical data on race, marital status, tumor stage, treatment methods, etc. Finally, a total of 8,997 patients were included and divided into the Training Group and the Testing Group.

### 2.2. Data Collection

Baseline variables including age, gender, race, marital status, the primary site of tumors, American Joint Committee on Cancer (AJCC) stage, TNM stage, tumor size, insurance situation, treatment methods (including surgery, radiotherapy, and chemotherapy), grade, vital status, the number of regional nodes positive, and follow-up time were collected.

### 2.3. Statistical Analysis

Based on the data from the Training Group, baseline variables were first included in the univariate analysis. The variables with statistical significance were then included in the multivariate Cox regression to explore prognostic factors associated with the overall survival of stomach cancer, and a nomogram was thereby developed. Subsequently, the data of the Testing Group were applied to externally validate the predictive effect of our nomogram.

All statistical tests were performed using the two-sided test, and *P* < 0.05 was considered statistically significant. The Kolmogorov–Smirnov (KS) test was used for the measurement data. Normally distributed data were described as mean ± standard deviation (Mean ± SD), and nonnormal data were described as median and quartile *M* (*Q*_1_, *Q*_3_). The enumeration data were described as the number of cases and constituent ratio *n* (%). Cox proportional hazards model was used in both univariate and multivariate analyses, where hazard ratios (HRs) and 95% confidence intervals (CIs) were determined. A nomogram was plotted according to the results of the multivariate Cox analysis. R version 4.0.2 (The R Foundation for Statistical Computing, Vienna, Austria) was used for plotting the nomogram, Kaplan–Meier (KM) curves, calibration curves, receiver operating characteristic (ROC) curve, and KS curve. KM curves were utilized to assess the survival of stomach cancer patients, in terms of age, races, marital status, TNM stages, chemotherapy, surgery, radiotherapy, grade, primary site, and tumor size. The discrimination of the nomogram for predicting the mortality was evaluated using ROC and KS curves. The agreement between the predicted and actual survival of patients was assessed by calibration curve.

## 3. Results

### 3.1. Baseline Characteristics

In the current study, 4,456 eligible patients including 2,557 males (57.38%) and 1,899 females (42.62%) were enrolled in the Training Group. Among them, 1,700 patients were <65 years (38.15%), 2,017 were between 65 and 80 years (45.26%), and 739 were >80 years (16.58%). For race, 2588 (57.41%) were whites, 726 (16.29%) were blacks, and 1,171 (26.30%) were others. About marital status, 2,722 (61.09%) were married, 663 (14.88%) were widowed, and 1,071 (24.04%) were others (single, divorced, separated, and unmarried). For insurance situation, 905 patients (20.31%) received Medicaid, 2,708 (60.77%) were insured, 694 (15.57%) had no specific insurance, and 149 (3.34%) were not insured. The primary sites of stomach cancer in patients included the fundus (*n* = 162, 3.68%), the body of stomach (*n* = 629, 14.12%), the antrum (*n* = 1,649, 37.01%), the pylorus (*n* = 228, 5.12%), the lesser curvature (*n* = 671, 15.06%), the greater curvature (*n* = 248, 5.57%), the overlapping lesion (*n* = 478, 10.73%), and the stomach or NOS (*n* = 389, 8.73%). The proportions of T4 stage, N3 stage, M1 stage, and tumor size >4 cm were 32.38% (*n* = 1,143), 23.65% (*n* = 1,054), 10.26% (*n* = 457), and 51.39% (*n* = 2,290), respectively. The number of patients with grade I, II, III, and IV were 236 (5.30%), 1,113 (24.98%), 3,001 (67.35%), and 106 (2.38%), respectively. For treatment methods, almost all patients (99.17%) received surgery; most of the patients (74.73%) did not receive radiotherapy; 2,245 patients (50.38%) received chemotherapy and 2,211 patients (49.62%) did not. The median number of regional nodes positive was 1 (0, 6), and the median follow-up time was 20.0 (11.0, 35.0) months. As for vital status, 2,461 patients (55.23%) were alive and 1,995 patients (44.77%) died during the follow-up period, with the longest follow-up time of 60 months.

Patients in the Testing Group showed similar characteristics to those in the Training Group. The baseline characteristics of the Training Group and the Testing Group are summarized in Table 1.

### 3.2. Univariate and Multivariate Analyses

By analyzing the five-year survival in the Training Group, the results suggested that compared with patients <65 years old, the mortality risk was 0.147-fold higher in patients between 65 and 80 years (HR = 1.147, 95% CI: 1.038–1.267) and 0.717-fold higher in those ≥81 years (HR = 1.717, 95% CI: 1.521–1.939). In contrast to White patients, patients of other races (including American Indian, Alaska Native, and Asian-Pacific Islander) had a 0.294-fold reduced mortality risk (HR = 0.706, 95% CI: 0.663–0.788). As regards marital status, the risk of death was 1.457 times higher in widowed patients than that in married patients (HR = 1.457, 95% CI: 1.293–1.643), and the risk was 1.150 times higher in patients with other marital status (including single, divorced, separated, and unmarried) (HR = 1.150, 95% CI: 1.034–1.277). Compared with patients with the unclear primary site, patients with the primary site of the body of the stomach had a 0.300-fold reduced risk of mortality (HR = 0.700, 95% CI: 0.581–0.843); patients with the primary site of the antrum had a 0.184-fold reduced risk (HR = 0.816, 95% CI: 0.698–0.953); and patients with the primary site of the lesser curvature had a 0.297-fold reduced risk (HR = 0.703, 95% CI: 0.586–0.843). Concerning tumor stage, as compared with patients at the T1 stage, the mortality risk was 1.439 times in patients at the T2 stage (HR = 1.439, 95% CI: 1.164–1.779), 2.903 times at T3 stage (HR = 2.903, 95% CI: 2.473–3.407), and 5.641 times at T4 stage (HR = 5.641, 95% CI: 4.832–6.586); in comparison with patients at N0 stage, the mortality risk was 2.031 times higher in patients at N1 stage (HR = 2.031, 95% CI: 1.769–2.330), 2.670 times higher at N2 stage (HR = 2.670, 95% CI: 2.337–3.052), and 4.310 times higher at N3 stage (HR = 4.310, 95% CI: 3.833–4.846); patients at M1 stage had a 3.196 times higher risk of mortality than those at M0 stage (HR = 3.196, 95% CI: 2.848–3.585). Patients with tumor >4 cm showed a 1.088 times (HR = 2.088, 95% CI: 1.905–2.289) higher mortality risk than patients with tumor ≤4 cm. With respect to treatment methods, patients without surgery had a 2.424-fold (HR = 3.424, 95% CI: 2.386–4.914) increased mortality risk than those with surgery; patients without radiotherapy had a 0.232-fold (HR = 1.232, 95% CI: 1.112–1.364) increased risk than those with radiotherapy; and patients without chemotherapy had a 0.184-fold (HR = 1.184, 95% CI: 1.084–1.293) increased risk than those with chemotherapy. The mortality risk increased 0.504-fold with one increase in the number of regional nodes positive (HR = 1.054, 95% CI: 1.049–1.058). Compared with grade I and II, cases with grade III and IV had a higher death risk (HR = 1.656, 95% CI: 1.492–1.837). There was no statistical difference in the risk of death between males and females (HR = 0.973, 95% CI: 0.890–1.064) (Table 2, Figures 1 and 2).

After the univariate analysis, statistically significant variables were included in the multivariate Cox regression for further analysis. The results showed that age, race, marital status, TNM stage, surgery, chemotherapy, grade, and regional nodes positive were all identified as independent prognostic factors for the survival of stomach cancer patients (Table 3).

### 3.3. Development and Validation of a Nomogram

Based on the results of the multivariate analysis, the nomogram was plotted (Figure 3). Take one case in the Training Group as an example, the patient was married and from other races, aged 70 years old. The patient had a tumor grade of III + IV and was at M1, N3, and T4 stages with 11 regional nodes positive. Also, the patient received surgery and chemotherapy. In our Cox model, the patients had a total score of 545 points, and the probability of survival longer than 20 months was 70.5%. The outcome for the patient was dead, confirming the accuracy of our model (Figure 4). The formula for prediction was *h* (*t*, *X*) = *h*_0_ (*t*) exp (0.290 (aged between 65 and 80 years) + 0.495 (age ≥81 years)–0.281 (other races) + 0.224 widowed + 0.140 (other marital status) + 0.320 *T*2 + 0.905 *T*3 + 1.379 *T*4 + 0.557 *N*1 + 0.668 *N*2 + 0.840 *N*3 + 0.660 M1–1.424 surgery–0.750 chemotherapy + 0.199 (tumor grade III + IV) + 0.017 (positive nodes).

The nomogram was then externally validated in the Testing Group. The concordance index (C-index) of the Training Group was 0.790 (95% CI: 0.777, 0.803), with the specificity of 0.717 (95% CI: 0.699, 0.735) and the sensitivity of 0.729 (95% CI: 0.709, 0.748). For the Testing Group, the C-index was 0.789 (95% CI: 0.776, 0.802), with the specificity of 0.713 (95% CI: 0.695, 0.731) and the sensitivity of 0.729 (95% CI: 0.710, 0.748) (Table 4). The ROC curves for predicting the mortality of patients with stomach cancer are shown in Figure 5(a), with the AUCs of 0.790 (95% CI: 0.777, 0.803) in the Training Group and 0.789 (95% CI: 0.776, 0.802) in the Testing Group. The KS curve was also drawn with the KS value of 0.45, indicating good discrimination of the nomogram (Figure 5(b)). Besides, the calibration curves of the Training Group and the Testing Group are shown in Figures 6(a) and 6(b), respectively, suggesting good agreement between the predicted survival of our nomogram and actual survival of patients.

## 4. Discussion

At present, stomach cancer is a very common cancer worldwide with a poor prognosis and long-term survival. In the current study, we developed a novel nomogram model to predict the overall survival of patients with stomach cancer. Variables including age, race, marital status, TNM stage, surgery, chemotherapy, tumor grade, and the number of regional nodes positive were significantly associated with the overall survival. As expected, our nomogram model showed good performance both in calibration and discrimination, with a C-index of 0.790 and a KS value of 0.45. Besides, the results of the external validation also confirmed the stability and accuracy of this nomogram.

Currently, the constructed nomogram includes several prognostic factors containing age, race, marital status, TNM stage, surgery, chemotherapy, tumor grade, and the number of regional nodes positive. Many studies have demonstrated that age is an important prognostic factor in the survival of cancer patients [7, 13–15]. Our results indicated that older age was associated with an increased risk of poor survival in patients with stomach cancer. Also, patients of non-White or non-Black races and those receiving surgery or chemotherapy showed lower mortality risks, which were all consistent with previous studies [14, 16]. A higher TNM stage and a higher tumor grade were also associated with worse survival. Besides, patients at the later TNM stage showed increased mortality risk. A possible explanation for this might be that quite a few patients with stomach cancer were already at a later stage at the time of diagnosis and never underwent surgery or chemotherapy before, which may increase the risk of recurrence or even death [17]. Besides, in a Chinese population-based study, T stage, number of metastatic lymph nodes, lymph node-positive rate, adjuvant chemotherapy, and diameter of the tumor were included in the nomogram [16]. In a Korean study, age, gender, tumor location, depth of invasion, number of positive lymph nodes, and number of examined lymph nodes were significantly associated with the overall survival [15]. However, according to our multivariate Cox regression, some variables such as gender, tumor size, and tumor location were not significantly associated with the overall survival. It might be speculated that the difference was due to different populations, which require multicenter studies for verification.

Over the past few decades, the AJCC staging system has become the most widely accepted and used classification system for stomach cancer. However, recent studies have proposed that the AJCC staging system ignored the biological heterogeneity of patients and was not sufficient to predict the recurrence of cancer, resulting in great differences in treatment effects even in patients with the same stage using the same treatment regimen [18–20]. To date, some studies have established nomograms to predict the overall survival of stomach cancer [7, 13, 14, 16, 21]. However, most of them were based on the patients who received surgical treatment, and patients who did not were excluded. The proposed nomogram also included patients who did not receive surgery or other treatment and set whether patients received surgery, chemotherapy, and radiotherapy or not as variables for analysis. At the same time, the prognostic factors in our nomogram were all available and easily collected in clinical practice. To further assess the performance of the nomogram model, the calibration, ROC, and KS curves were plotted. The nomogram showed good discrimination with a C-index of 0.790 and a KS value of 0.45 for the training set. Moreover, external validation was also performed, and the C-index of 0.789 for the testing set confirmed the good performance of our nomogram.

However, there are still some limitations in our study. Although we selected the patient data from 2012–2016 for external validation, the data were all derived from the SEER database, which is mainly composed of the American population with limited universal applicability. For special medical images, the treatments involve not only regional assessments and surgical planning but also segmentation and thickness computation [22–25]. In addition, the SEER database is an open data platform, which collects data on patient demographics, primary tumor site, tumor morphology, stage at diagnosis, and first course of treatment, and patients were followed up for vital status. The potential factors including rural or urban areas and physical health (such as height, weight, and diet) that could affect the survival of stomach cancer patients were not recorded in the database, so further studies should be conducted to improve the nomogram. In the future, the results of the study would be more accurate if our nomogram was externally validated in other cohorts including more populations within the same period.

## 5. Conclusion

In the present study, we have developed an effective nomogram with ten easily acquired prognostic factors including age, race, marital status, TNM stage, surgery, chemotherapy, tumor grade, and the number of regional nodes positive. The nomogram could accurately predict the overall survival of patients with stomach cancer and performed well on external validation. We expect that the nomogram would be helpful for both patients and clinicians to improve the individualized survival prediction and decision-making, thereby improving the outcome and survival of stomach cancer.

## Figures and Tables

**Figure 1:** Kaplan–Meier curves for survival in stomach cancer patients regarding (a) different age, (b) races, (c) marital status, and (d) T, (e) N, and (f) M stages.

**Figure 2:** Kaplan–Meier curves for survival in stomach cancer patients regarding (a) chemotherapy, (b) surgery, (c) radiation, (d) grade, (e) primary site, and (f) tumor size.

**Figure 3:** Nomogram for predicting survival probability in stomach cancer.

**Figure 4:** Example of the nomogram for predicting the individual survival probability in stomach cancer.

**Figure 5:** (a) ROC curve and (b) KS curve for the Training Group.

**Figure 6:** Calibration curves for the (a) Training Group and (b) the Testing Group.

**Table 1:** Baseline characteristics of the Training Group and the Testing Group.

Variables	Training Group (*n* = 4456)	Testing Group (*n* = 4541)
Age, years, *n* (%)		
<65	1700 (38.15)	1735 (38.21)
65–80	2017 (45.26)	2059 (45.34)
≥81	739 (16.58)	747 (16.45)
Gender, *n* (%)		
Male	2557 (57.38)	2600 (57.26)
Female	1899 (42.62)	1941 (42.74)
Race, *n* (%)		
White	2558 (57.41)	2612 (57.52)
Black	726 (16.29)	737 (16.23)
Others	1172 (26.30)	1192 (26.25)
Marital status, *n* (%)		
Married	2722 (61.09)	2775 (61.11)
Widowed	663 (14.88)	673 (14.82)
Others	1071 (24.04)	1093 (24.07)
Primary site, *n* (%)		
Fundus	164 (3.68)	166 (3.66)
Body of stomach	629 (14.12)	641 (14.12)
Antrum	1649 (37.01)	1673 (36.84)
Pylorus	228 (5.12)	236 (5.20)
Lesser curvature	671 (15.06)	685 (15.08)
Greater curvature	248 (5.57)	255 (5.62)
Overlapping lesion	478 (10.73)	487 (10.72)
Stomach or NOS	389 (8.73)	398 (8.76)
AJCC stage, *n* (%)		
I	1223 (27.45)	1232 (27.13)
II	1144 (25.67)	1168 (25.72)
III	1632 (36.62)	1677 (36.93)
IV	457 (10.26)	464 (10.22)
T stage, *n* (%)		
T1	997 (22.37)	1008 (22.20)
T2	580 (13.02)	586 (12.90)
T3	1436 (32.23)	1465 (32.26)
T4	1443 (32.38)	1482 (32.64)
N stage, *n* (%)		
N0	1785 (40.06)	1801 (39.66)
N1	825 (18.51)	847 (18.65)
N2	792 (17.77)	811 (17.86)
N3	1054 (23.65)	1082 (23.83)
M stage, *n* (%)		
M0	3999 (89.74)	4077 (89.78)
M1	457 (10.26)	464 (10.22)
Tumor size, cm, *n* (%)		
≤4	2166 (48.61)	2209 (48.65)
>4	2290 (51.39)	2332 (51.35)
Insurance, *n* (%)		
Any Medicaid	905 (20.31)	929 (20.46)
Insured	2708 (60.77)	2755 (60.67)
No specific insured	694 (15.57)	707 (15.57)
Uninsured	149 (3.34)	150 (3.30)
Surgery, *n* (%)		
Yes	4419 (99.17)	4503 (99.16)
No	37 (0.83)	38 (0.84)
Radiation, *n* (%)		
Yes	1126 (25.27)	1214 (26.73)
No	3330 (74.73)	3327 (73.27)
Chemotherapy, *n* (%)		
Yes	2245 (50.38)	2288 (50.39)
No	2211 (49.62)	2253 (49.61)
Grade, *n* (%)		
I	236 (5.30)	239 (5.26)
II	1113 (24.98)	1137 (25.04)
III	3001 (67.35)	3057 (67.32)
IV	106 (2.38)	108 (2.38)
Vital status, *n* (%)		
Alive	2461 (55.23)	2508 (55.23)
Dead	1995 (44.77)	2033 (44.77)
Regional nodes positive (M (*Q*_1_, *Q*_3_))	1 (0, 6)	1 (0, 6)
Follow-up time, months (M (*Q*_1_, *Q*_3_))	20.0 (11.0, 35.0)	20.0 (11.0, 35.0)

NOS, not otherwise specified; AJCC, American Joint Committee on Cancer.

**Table 2:** Univariate analysis of survival in the Training Group.

Variables	Training Group (*n* = 4456)			
	5-year survival (%)	HR	95% CI	*P* value
Age, years				
<65	60.00	Ref		
65–80	55.78	1.147	(1.038, 1.267)	0.007
≥81	42.76	1.717	(1.521, 1.939)	<0.001
Gender				
Male	54.91	Ref		
Female	55.66	0.973	(0.890, 1.064)	0.549
Race				
White	52.11	Ref		
Black	53.72	0.952	(0.844, 1.074)	0.427
Others	62.97	0.706	(0.663, 0.788)	<0.001
Marital status				
Married	57.71	Ref		
Widowed	47.21	1.457	(1.293, 1.643)	<0.001
Others	53.87	1.150	(1.034, 1.277)	0.010
Primary site				
Stomach, NOS	48.07	Ref		
Fundus	56.10	0.824	(0.629, 1.078)	0.158
Body of stomach	60.73	0.700	(0.581, 0.843)	<0.001
Antrum	55.61	0.816	(0.698, 0.953)	0.010
Pylorus	57.02	0.829	(0.651, 1.055)	0.127
Lesser curvature	59.62	0.703	(0.586, 0.843)	<0.001
Greater curvature	54.84	0.831	(0.659, 1.046)	0.115
Overlapping lesion	45.40	1.083	(0.901, 1.301)	0.395
T stage				
T1	80.54	Ref		
T2	73.62	1.439	(1.164, 1.779)	<0.001
T3	71.17	2.903	(2.473, 3.407)	<0.001
T4	31.46	5.641	(4.832, 6.586)	<0.001
N stage				
N0	74.51	Ref		
N1	55.39	2.031	(1.769, 2.330)	<0.001
N2	47.73	2.670	(2.337, 3.052)	<0.001
N3	47.47	4.310	(3.833, 4.846)	<0.001
M stage				
M0	59.19	Ref		
M1	20.57	3.196	(2.848, 3.585)	<0.001
Tumor size, cm				
≤4	67.44	Ref		
>4	77.33	2.088	(1.905, 2.289)	<0.001
Insurance				
Uninsured	54.36	Ref		
Any Medicaid	53.15	0.933	(0.719, 1.212)	0.603
Insured	56.61	0.985	(0.762, 1.272)	0.908
No specific insured	52.74	0.826	(0.647, 1.054)	0.125
Surgery				
Yes	55.53	Ref		
No	18.92	3.424	(2.386, 4.914)	<0.001
Radiation				
Yes	56.75	Ref		
No	55.71	1.232	(1.112, 1.364)	<0.001
Chemotherapy				
Yes	80.08	Ref		
No	54.68	1.184	(1.084, 1.293)	<0.001
Grade				
I + II	65.75	Ref		
III + IV	50.66	1.656	(1.492, 1.837)	<0.001
Regional nodes positive (M (*Q*1, *Q*3))	1.054		(1.049, 1.058)	<0.001

HR, hazard ratio; CI, confidence interval; NOS, not otherwise specified; AJCC, American Joint Committee on Cancer.

**Table 3:** Multivariate analysis of survival in the Training Group.

Variables	Training Group (*n* = 4456)		
	HR	95% CI	*P* value
Age, years			
<65	Ref		
65–80	1.337	(1.203, 1.486)	<0.001
≥81	1.640	(1.424, 1.888)	<0.001
Race			
White	Ref		
Black	1.125	(0.994, 1.274)	0.062
Others	0.755	(0.677, 0.843)	<0.001
Marital status			
Married	Ref		
Widowed	1.252	(1.103, 1.420)	0.001
Others	1.150	(1.032, 1.281)	0.011
T stage			
T1	Ref		
T2	1.377	(1.109, 1.710)	0.004
T3	2.473	(2.074, 2.949)	<0.001
T4	3.971	(3.315, 4.756)	<0.001
N stage			
N0	Ref		
N1	1.746	(1.504, 2.026)	<0.001
N2	1.951	(1.676, 2.271)	<0.001
N3	2.316	(1.928, 2.783)	<0.001
M stage			
M0	Ref		
M1	1.934	(1.716, 2.181)	<0.001
Surgery			
No	Ref		
Yes	0.241	(0.167, 0.346)	<0.001
Chemotherapy			
No	Ref		
Yes	0.473	(0.427, 0.523)	<0.001
Grade			
I + II	Ref		
III + IV	1.220	(1.093, 1.362)	<0.001
Regional nodes positive	1.017	(1.009, 1.026)	<0.001

HR, hazard ratio; CI, confidence interval.

**Table 4:** Discrimination of the nomogram.

Variables (95% CI)	Training Group	Testing Group
C-index	0.790 (0.777, 0.803)	0.789 (0.776, 0.802)
Accuracy	0.722 (0.709, 0.736)	0.720 (0.707, 0.733)
Specificity	0.717 (0.699, 0.735)	0.713 (0.695, 0.731)
Sensitivity	0.729 (0.709, 0.748)	0.729 (0.710, 0.748)
PPV	0.676 (0.657, 0.737)	0.673 (0.653, 0.733)
NPV	0.765 (0.748, 0.783)	0.764 (0.747, 0.782)

CI, confidence interval; PPV, positive predictive value; NPV, negative predictive value.

## Data Availability

The data utilized to support the findings are available from the corresponding authors upon request.

## References

[1] Gao J.-P., Xu W., Liu W.-T., Yan M., Zhu Z.-G. (2018). Tumor heterogeneity of gastric cancer: from the perspective of tumor-initiating cell. *World Journal of Gastroenterology*.

[2] Bray F., Ferlay J., Soerjomataram I., Siegel R. L., Torre L. A., Jemal A. (2018). Global cancer statistics 2018: GLOBOCAN estimates of incidence and mortality worldwide for 36 cancers in 185 countries. *CA: A Cancer Journal for Clinicians*.

[3] Poorolajal J., Moradi L., Mohammadi Y., Cheraghi Z., Gohari-Ensaf F. (2020). Risk factors for stomach cancer: a systematic review and meta-analysis. *Epidemiology and Health*.

[4] Sung H., Ferlay J., Siegel R. L. (2021). Global cancer statistics 2020: GLOBOCAN estimates of incidence and mortality worldwide for 36 cancers in 185 countries. *CA: A Cancer Journal for Clinicians*.

[5] Reim D., Loos M., Vogl F. (2013). Prognostic implications of the seventh edition of the international union against cancer classification for patients with gastric cancer: the Western experience of patients treated in a single-center European institution. *Journal of Clinical Oncology*.

[6] Ajani J. A., Lee J., Sano T., Janjigian Y. Y., Fan D., Song S. (2017). Gastric adenocarcinoma. *Nature Reviews Disease Primers*.

[7] Zheng Z.-F., Lu J., Wang W. (2018). Development and external validation of a simplified nomogram predicting individual survival after R0 resection for gastric cancer: an international, multicenter study. *Annals of Surgical Oncology*.

[8] Kattan M. W., Zelefsky M. J., Kupelian P. A. (2003). Pretreatment nomogram that predicts 5-year probability of metastasis following three-dimensional conformal radiation therapy for localized prostate cancer. *Journal of Clinical Oncology*.

[9] Marko N. F., Xu Z., Gao T., Kattan M. W., Weil R. J. (2012). Predicting survival in women with breast cancer and brain metastasis. *Cancer*.

[10] Amer K. M., Munn M., Congiusta D., Abraham J. A., Basu Mallick A. (2020). Survival and prognosis of chondrosarcoma subtypes: SEER database analysis. *Journal of Orthopaedic Research*.

[11] Kim S. Y., Yoon M. J., Park Y. I., Kim M. J., Nam B.-H., Park S. R. (2018). Nomograms predicting survival of patients with unresectable or metastatic gastric cancer who receive combination cytotoxic chemotherapy as first-line treatment. *Gastric Cancer*.

[12] Shi H., Jiang Y., Cao H., Zhu H., Chen B., Ji W. (2018). Nomogram based on systemic immune-inflammation index to predict overall survival in gastric cancer patients. *Disease Markers*.

[13] Bando E., Ji X., Kattan M. W. (2020). Development and validation of a pretreatment nomogram to predict overall survival in gastric cancer. *Cancer Medicine*.

[14] Wang C.-Y., Yang J., Zi H. (2020). Nomogram for predicting the survival of gastric adenocarcinoma patients who receive surgery and chemotherapy. *BMC Cancer*.

[15] Han D.-S., Suh Y.-S., Kong S.-H. (2012). Nomogram predicting long-term survival after d2 gastrectomy for gastric cancer. *Journal of Clinical Oncology*.

[16] Zhang P. F., Du Z. D., Wen F. (2020). Development and validation of a nomogram for predicting overall survival of gastric cancer patients after D2R0 resection. *European Journal of Cancer Care*.

[17] Spolverato G., Ejaz A., Kim Y. (2014). Rates and patterns of recurrence after curative intent resection for gastric cancer: a United States multi-institutional analysis. *Journal of the American College of Surgeons*.

[18] Dikken J. L., van de Velde C. J. H., Gönen M., Verheij M., Brennan M. F., Coit D. G. (2012). The New American Joint Committee on Cancer/International Union against Cancer staging system for adenocarcinoma of the stomach: increased complexity without clear improvement in predictive accuracy. *Annals of Surgical Oncology*.

[19] Yoon H. M., Ryu K. W., Nam B. H. (2012). Is the new seventh AJCC/UICC staging system appropriate for patients with gastric cancer?. *Journal of the American College of Surgeons*.

[20] Marrelli D., Morgagni P., de Manzoni G. (2012). Prognostic value of the 7th AJCC/UICC TNM classification of n gastric cancer. *Annals of Surgery*.

[21] Woo Y., Son T., Song K. (2016). A novel prediction model of prognosis after gastrectomy for gastric carcinoma. *Annals of Surgery*.

[22] Faisal A., Ng S.-C., Goh S.-L., Lai K. W. (2018). Knee cartilage segmentation and thickness computation from ultrasound images. *Medical, & Biological Engineering & Computing*.

[23] Jahanzad Z., Liew Y. M., Bilgen M. (2015). Regional assessment of LV wall in infarcted heart using tagged MRI and cardiac modelling. *Physics in Medicine and Biology*.

[24] Chai H., Wee L., Swee T., Salleh S.-H., Chea L. (2011). An artifacts removal post-processing for epiphyseal region-of-interest (EROI) localization in automated bone age assessment (BAA). *BioMedical Engineering Online*.

[25] Khalil A., Faisal A., Ng S. C., Liew Y. M., Lai K. W. (2017). Multimodality registration of two-dimensional echocardiography and cardiac CT for mitral valve diagnosis and surgical planning. *Journal of Medical Imaging*.

